This article has been retracted.

# Exosome-transmitted miR-128-3p increase chemosensitivity of oxaliplatin-resistant colorectal cancer

**DOI:** 10.1186/s12943-019-0981-7

**Published:** 2019-03-19

**Authors:** Tong Liu, Xin Zhang, Lutao Du, Yunshan Wang, Xiaoming Liu, Hui Tian, Lili Wang, Peilong Li, Yinghui Zhao, Weili Duan, Yujiao Xie, Zhaowei Sun, Chuanxin Wang

**Affiliations:** 1 Department of Clinical Laboratory, The Second Hospital of Shandong University, No. 247 Beiyuan Street, Jinan, 250033 China; 2 Department of Clinical Laboratory, Qilu Hospital, Shandong University, Jinan, 250012 Shandong Province China; 3 Department of Preventive Medicine, Shandong Provincial Traditional Chinese Medical Hospital, Jinan, 250012 People’s Republic of China; 4 Cancer Center, Qilu Hospital, Shandong University, Jinan, 250012 Shandong Province China; 5 Department of Surgery, The Affiliated Hospital of Medical College Qingdao University, Qingdao, 266071 Shandong Province China

**Keywords:** miR-218-3p, Exosome, Colorectal cancer, Chemoresistance, Epithelial-mesenchymal transition, Drug efflux

## Abstract

**Background:**

Oxaliplatin resistance is a major challenge for treatment of advanced colorectal cancer (CRC). Both acquisition of epithelial-mesenchymal transition (EMT) and suppressed drug accumulation in cancer cells contributes to development of oxaliplatin resistance. Aberrant expression of small noncoding RNA, miR-128-3p, has been shown to be a key regulator in tumorigenesis and cancer development. However, its roles in the progression of CRC and oxaliplatin-resistance are largely unknown.

**Methods:**

Oxaliplatin-resistant CRC and normal intestinal FHC cells were transfected with a miR-128-3p expression lentivirus. After transfection, FHC-derived exosomes were isolated and co-cultured with CRC cells. miR-128-3p expression in resistant CRC cells, FHC cells, and exosomes was quantified by quantitative real-time PCR (RT-qPCR). The mRNA and protein levels of miR-128-3p target genes in resistant CRC cells were quantified by RT-qPCR and western blot, respectively. The effects of miR-128-3p on CRC cell viability, apoptosis, EMT, motility and drug efflux were evaluated by CCK8, flow cytometry, Transwell and wound healing assays, immunofluorescence, and atomic absorption spectrophotometry. Xenograft models were used to determine whether miR-128-3p loaded exosomes can re-sensitize CRC cells to oxaliplatin in vivo.

**Results:**

In our established stable oxaliplatin-resistant CRC cell lines, in vitro and vivo studies revealed miR-128-3p suppressed EMT and increased intracellular oxaliplatin accumulation. Importantly, our results indicated that lower miR-128-3p expression was associated with poor oxaliplatin response in advanced human CRC patients. Moreover, data showed that miR-128-3p-transfected FHC cells effectively packaged miR-128-3p into secreted exosomes and mediated miR-128-3p delivery to oxaliplatin-resistant cells, improving oxaliplatin response in CRC cells both in vitro and in vivo. In addition, miR-128-3p overexpression up-regulated E-cadherin levels and inhibited oxaliplatin-induced EMT by suppressing Bmi1 expression in resistant cells. Meanwhile, it also decreased oxaliplatin efflux through suppressed expression of the drug transporter MRP5.

**Conclusion:**

Our results demonstrate that miR-128-3p delivery via exosomes represents a novel strategy enhancing chemosensitivity in CRC through negative regulation of Bmi1 and MRP5. Moreover, miR-128-3p may be a promising diagnostic and prognostic marker for oxaliplatin-based chemotherapy.

**Electronic supplementary material:**

The online version of this article (10.1186/s12943-019-0981-7) contains supplementary material, which is available to authorized users.

## Background

The global incidence of colorectal cancer (CRC) is increasing; annually, more than 1.2 million new cases of CRC are diagnosed and 608,700 deaths have been attributed to this disease [1]. Oxaliplatin is one of the most commonly used chemotherapeutics following surgical resection, especially for patients with stage II and stage III disease [2]. Oxaliplatin causes intrastrand and interstrand DNA-platinum adducts and then inhibit gene transcription by segregation of transcription factors or lead to G2/M stage arrest. Moreover, the apoptotic cascade initiated by oxaliplatin is characterized by translocation of Bax to the mitochondria, cytochrome c release into the cytosol and caspase 3 activation [3]. Unfortunately, de novo and acquired oxaliplatin resistance remains a major challenge in CRC treatment [4]. The development of resistance is multi-factorial, including: up-regulation of ATP-binding cassette transporters (decreasing drug penetrance), over-active DNA damage response, enhanced anti-apoptosis, and epithelial-to-mesenchymal transition (EMT) [5–7]. Therefore, elucidating the underlying mechanisms and developing effective strategies against oxaliplatin resistance are clinical priorities.

MiR-128-3p, as a microRNA, negatively correlates with MET expression in breast cancer and inhibits hepatocyte growth factor-induced cell migration by directly targeting MET [8]. Previous microarray studies revealed that miR-128-3p expression was decreased in adenocarcinoma or metastatic prostate cancer when compared to normal/benign prostate tissues [9, 10]. Subsequent studies reported that miR-128-3p expression levels were an independent prognostic marker that played important roles in cell proliferation, metabolism, and metastasis (lung, breast, glioblastoma, gastric cancer, and CRC) [11–15]. Although these findings support the notion that aberrant miR-128-3p expression is involved in several important tumorigenic molecular pathways, the role of miR-128-3p in oxaliplatin resistance observed in advanced CRC remains to be elucidated.

Exosomes were described in as 40–150 nm diameter vesicles secreted from several mammalian cell types [16]. Exosomes can dock and fuse to the membrane of target-cells, delivering exosomal surface proteins and cytoplasm [17, 18]. There is growing interest in utilizing exosomes as in vivo delivery vehicles for miRNA as exosomes do not elicit adverse immune responses and possess low-risk for tumor formation [19]. Furthermore, exosomes loaded with therapeutic miRNAs can be manufactured in bulk by exosome producing cells in vitro thus enabling personalized treatment [20]. These findings provide rationale for designing an exosome-based therapeutic strategy for targeting oxaliplatin-resistant CRC. Here, we investigate the utility of miR-128-3p as a prognostic marker and its potential role in transcriptional regulation in CRC patients receiving oxaliplatin. Furthermore, we explore a novel exosome-based delivery of miR-128-3p as a therapeutic strategy for miR-128-3p-mediated chemotherapy sensitization.

## Methods

### Cell culture

All cell lines were purchased from Type Culture Collection of the Chinese Academy of Sciences (Shanghai, China). Oxaliplatin (Sanofi-Synthelabo, NY, USA) was purchased from the Second Hospital of Shandong University. Oxaliplatin-resistant cell lines (HCT116OxR and HT29OxR) were established as previously described [2, 21, 22]. For exosome co-cultures, 1 μg/ml (as determined by BCA protein assay (Thermo Fisher Scientific, USA)) of exosomes were added to the culture medium of recipient cells (5 × 10^6^).

### Clinical CRC patient samples

Tissue samples were collected prior to initiation of oxaliplatin therapy from surgical specimens or biopsies of advanced CRC patients and obtained informed consent from the Second Hospital of Shandong University (*n* = 86), Qilu Hospital of Shandong University (*n* = 67) and Shandong Provincial Traditional Chinese Medical Hospital (*n* = 20) between July 2008 and February 2018. This study was approved by the Ethics Committee of the Second Hospital of Shandong University. Patients in the oxaliplatin group were treated with at least six cycles of oxaliplatin, while patients in untreated group received no chemotherapy or stopped oxaliplatin therapy (< 21 days) due to adverse effects. Detailed clinical characteristics of patients in training phase are listed in Additional file 1: Table S1.

Tumor response to chemotherapy was assessed as a 3-dimensional volume reduction rate or tumor response rate (radiologic assessment), and evaluated as per the Response Evaluation Criteria in Solid Tumors (RECIST) guidelines [23]. Patients with symptomatic deterioration, or appearance of new lesions, or radiologic assessment of ≥25% tumor regrowth in validation phase were allocated to the progressed disease (PD) group (*n* = 35) and remaining to non-PD group (*n* = 40). PFS was defined as the duration from tumor resection to PD. All patients were followed up in the clinic every 3 months (0–2 years), 6 months (2–4 years), and yearly until death or February 2018. Follow-up studies included computed tomography of the abdomen and postsurgical physical examination.

### Exosome purification and identification

Exosomes were isolated from FHC cell conditioned medium by 0.22 μm filtration and ultracentrifugation as we previously described [24]. Transmission electron microscopy (JEM-1-11 microscope, Japan) was used to image exosomes at 100 keV, and quantified by Nanosight NS300 instrument (Malvern Instruments Ltd. UK) equipped with NTA 3.0 analytical software (Malvern Instruments Ltd. UK).

### Immunohistochemistry

Immunohistochemistry was done as previously reported [22]. Positive cells were counted in five random fields per slide. Interpretation of staining intensity of Bmi1 or MRP5 was made independently by two specialists, as no staining = 0, weak staining = 1 (1–25%), moderate staining = 2 (26–50%), and strong staining = 3 (51–100%).

### Quantitative real-time PCR

Cellular and exosomal RNAs were isolated using the miRNeasy Micro Kit (QIAGEN, Valencia, CA, USA). First-strand cDNA was synthesized with random primers using High Capacity cDNA Reverse Transcription Kit (Takara, Dalian, China). qPCR was performed using Power SYBR Green (Takara, Dalian, China) on a CFX96 Real-Time PCR Detection System (Bio-Rad, USA). Data was collected and normalized to U6 levels (for cellular miR-128-3p), GAPDH (for cellular Bmi1 and MRP5 mRNA) or miR-16 (for exosomal miR-128-3p) [25]. MicroRNA primers were synthesized by Ribobio (Guangzhou, China). mRNA primers are listed in Additional file 2: Table S3.

### Western blotting

Total protein of cells or exosomes was extracted with RIPA buffer (Sigma-Aldrich) and quantified with the BCA assay (Pierce, Rockford, IL), and Western Blot preformed as previously described [21]. Protein band intensity was quantified by densitometry using Image Lab software (Bio-Rad, Hercules, CA, USA). All antibodies used are shown in Additional file 3: Table S2.

### Lentiviral, plasmid and microRNA mimics package and cell transfection

Lentiviral plasmids encoding miR-128-3p and negative control were designed and produced by HANBIO (Shanghai, China). HCT116OxR and HT29OxR cells were transfected with lentivirus (pHB-U6-MCS-CMV-ZsGreen-PGK-PURO) at a multiplicity of infection (MOI) of 20 and 15, respectively. The cells were then selected with 1 μg/ml puromycin for 3 days. pcDNA3.1 vector containing Bmi1-wt, Bmi1-mut, MRP5-wt or MRP5-mut and control were purchased from GENECHEM (Shanghai, China). miR-128-3p mimics, inhibitor and control were produced by GENECHEM (Shanghai, China). Plasmid, mimics, inhibitor and negative control were transfected using Lipofectamine2000 (Invitrogen, California, USA) according to the manufacturer’s instructions.

### Cell viability assay

Cells viability was determined by Cell Counting Kit 8 (Dojindo, Japan) and measured at OD450 nm with the Thermo Scientific Multiskan FC (Thermo Fisher Scientific Corporation, USA).

### Cell migration and invasion assay

Cell migration was measured with Transwell assays, briefly cancer cells (2 × 10^4^ cells/well) were divided into different groups and seeded in the upper chambers in serum-free media with or without the Matrigel membrane. Meanwhile the lower chambers were loaded with RPMI1640 containing 5% FBS. After incubation at 37 °C, 5% CO_2_ for 24 h, the lower chamber was imaged using an inverted microscope. The upper chamber was cleaned with a cotton swab and the lower chamber was immersed and washed with PBS, fixed with 4% paraformaldehyde, stained with 0.1% crystal violet, washed three times with water, and imaged by Inversion Microscope (Zeiss, Germany).

### Animal experiments

Four-weeks old male BALB/C nude mice were purchased from Weitonglihua (Peking, China). HCT116OxR cells (5 × 10^6^ cells per mouse) were injected subcutaneously into the right flank of nude mice. Two weeks later, the nude mice generated tumors approximately 200 mm^3^ in size. Purified exosomes (5 μg) or PBS was then injected intratumorally twice weekly with or without oxaliplatin treatment (90 mg/m^2^). The tumor size and bodyweight were measured twice per week. After seven weeks, mice were sacrificed and tumor tissues were prepared for histological examination. Tumor volume (mm^3^) = 0.5 × width^2^ × length. All animal work was performed according to the Health guidelines, and protocols were approved by the Institutional Animal Care and Use Committee of Shandong University.

### Fluorescence assay

PKH67 (Sigma-Aldrich, USA) (1 μM) was used to label exosomes according to manufacturer’s instructions. 24 h after PKH67-labeled exosomes were incubated with HCT116OxR, 4′,6-diamidino-2-phenylindole (DAPI) (Invitrogen, USA) was used for cell nuclear staining. The slides were fluorescently visualized with a laser scanning microscope Axio-Imager-LSM800 (ZEISS, Germany). Rhodamine-conjugated secondary antibody (Cell Signaling Technology, USA) for γ-H_2_AX protein and DAPI for nuclear staining. The slides were visualized for immunofluorescence with a laser scanning microscope (Zeiss, Germany).

### Electroporation of miR-128-3p into exosomes

Gene Pulser X Electroporator (Bio-Rad, USA) was used to electroporate miR-128-3p into exosomes as previously described [22, 26, 27]. Briefly, 2 μg exosomes and 400 nmol miR-128-3p mimics were mixed in 400 μl of electroporation buffer at 4 °C. After electroporation at 350 V and 150 μF, the mixture was incubated at 37 °C for 30 mins to fully recover the membrane of exosomes.

### Luciferase reporter assay

Cells were co-transfected with Dual-Luciferase reporter system using pmiR-REPORT™ luciferase vectors containing wild-type or mutant 3`-UTR of Bmi1 and MRP5 and miR-128-3p mimics or miR-128-3p mimic-NC using Lipofectamine 2000 (Invitrogen, California, USA). Luciferase activity was measured by Dual-Luciferase Reporter Assay System (Beyotime Biotechnology, Shanghai, China) 48 h after transfection. Each group was run in triplicate in 24-well plates.

### Total cellular oxaliplatin and DNA-bound Pt assay

Intracellular Pt content was quantified as described previously [28]. Briefly, after treatment with oxaliplatin (30 μM), cells were lysed overnight with 0.1% triton-X-100 and 0.2% nitric acid. Cell lysates were subject to Atomic Absorption Spectrophotometry AA-6880 (SHIMADZU, Japan) and protein concentration was determined by BCA protein assay. DNA was isolated using DNeasy Blood & Tissue Kits (Qiagen, Valencia, CA) according to specifications and quantified with a NanoDrop spectrophotometer (Thermo Fisher Scientifc, USA). The same DNA hydrolysate was used for Pt measurements by Atomic Absorption Spectrophotometry AA-6880 (SHIMADZU, Japan).

### Statistical analysis

SPSS 17.0 for Windows (IBM Corporation, Armonk, NY) and GraphPad Prism (GraphPad Software, Inc., San Diego, CA, USA) software were used for statistical analyses. Statistical evaluations were determined using Student’s t-test (two-tailed), Kruskal–Wallis test or Spearman correlation test. Survival rates were calculated using the Kaplan–Meier method and comparisons were performed using the Log-rank test. The prognostic value was further verified using the Cox proportional hazards regression model. *P*- value of 0.05 or less was considered as statistically significant.

## Results

### Acquisition of oxaliplatin resistance induces EMT and enhances drug efflux in CRC cells

To obtain oxaliplatin-resistant colorectal cancer cells, we treated HCT116 and HT29 (lowest IC50 of seven CRC cell lines to oxaliplatin, Additional file 4: Figure S1A) in vitro with escalating oxaliplatin concentrations and then grafted cells into nude mice and performed cycles of oxaliplatin treatment along with three passages in vivo. CRC cells from the third passage xenografts that acquired oxaliplatin resistance at over clinically relevant concentrations (2 μM) [2] were named HCT116OxR and HT29OxR (Fig. 1a). Compared to parental cells, HCT116OxR and HT29OxR cells responded poorly to oxaliplatin, as illustrated by an increased IC50 and decreased drug-induced apoptosis (Fig. 1b, c and Additional file 4: Figure S1B). Meanwhile, resistant cells had phenotypic changes including: loss of intercellular adhesion, spindle-cell morphology (loss of cell polarity), and increased pseudopodia formation (Fig. 1d). Furthermore, resistant cells exhibited higher migration and invasion than their parental cells (Fig. 1e) and enhanced motility as observed in wound healing assay (Fig. 1f). Western blot analysis of resistant cells revealed typical of changes in cells with chemotherapy-induced EMT including decreased E-cadherin protein expression but dramatically increased N-cadherin, vimentin and fibronectin (Fig. 1g). In addition, quantitative platinum (Pt) analysis following oxaliplatin treatment (30 μM) for 24 h showed total intracellular Pt and DNA-bound Pt was lower in resistant than parental cells (Fig. 1h and i). Immunofluorescence assay using nuclear foci of γ-H_2_AX expression as an indicator of DNA double-strand breaks revealed that oxaliplatin induced more DNA damage in parental cells than oxaliplatin-resistant cells (Fig. 1j).

**Fig. 1:** Oxaliplatin-resistant HCT116OxR and HT29OxR cells have undergone EMT and increased drug efflux. **a** Schematic model presenting the process to acquire oxaliplatin-resistant CRC cells. **b** CCK8 assay of parent and resistant cell lines followed by oxaliplatin treatment at indicated concentrations. **c** Flow cytometry for apoptosis assay of parental and resistance cells with oxaliplatin treatment (30 μM). **d** The morphology of HCT116, HCT116-OxR, HT29 and HT29OxR cells. Scale bars, 50 μm. **e** Migration and invasion ability of parental and resistance CRC cells were assessed by Transwell assay. **f** Motility ability of parental and resistance CRC cells were assessed by wound healing assays. **g** Western blot analysis of protein E-cadherin (E-cad), N-cadherin (N-cad), Vimentin (Vim) and Fibronectin (Fn) expression in parental and resistance CRC cells. **h** Accumulation of Pt in parental and resistance cells following exposure to 30 μM, 24 h oxaliplatin treatment. **i** Total Pt-DNA adduct levels in parental and resistance cells following exposure to 30 μM, 24 h oxaliplatin treatment. **j** The immunofluorescence analysis of nuclear foci for γ-H_2_AX expression induced by oxaliplatin in parent and resistant cells after 24 h` oxaliplatin exposure. Scale bars, 10 μm. Results are presented as mean ± SD. *P < 0.05, **P < 0.01, ***P < 0.001

### Decreased expression of miR-128-3p is required for CRC oxaliplatin-resistance

Using RT-qPCR, we found all seven CRC cell lines expressed lower miR-128-3p than normal intestinal epithelial FHC cells (Additional file 4: Figure S1C). Importantly, miR-128-3p expression levels were also markedly higher expressed in HCT116 and HT29 compared with other CRC cell lines (Additional file 4: Figure S1C). Additionally, miR-128-3p expression was significantly decreased in resistant cells compared to respective parental cells (Fig. 2a). To further elucidate the role of miR-128-3p in oxaliplatin resistance, we stably overexpressed miR-128-3p using a lentiviral vector expression system (lenti-miR-128-3p) in oxaliplatin-resistant CRC cells. As expected, resistant cells transfected with lenti-miR-128-3p showed miR-128-3p levels several orders of magnitude higher than lenti-negative control (lenti-NC) transfected cells (Fig. 2b and Additional file 4: Figure S1D). Enhanced miR-128-3p expression in resistant cells reduced IC50 and increased cell apoptosis following oxaliplatin treatment (Fig. 2c, d and Additional file 4: Figure S1E–G). miR-128-3p overexpression significantly upregulated E-cadherin expression and downregulated N-cadherin, vimentin, and fibronectin expression in resistant cells (Fig. 2e and Additional file 4: Figure S1H–J). Moreover, miR-128-3p inhibited the migration, invasiveness, and motility of resistant cell lines (Fig. 2f, g Additional file 5: Figure S2A, B). Importantly, we found miR-128-3p downregulates drug efflux in CRC cells. Quantitative Pt analysis showed that following a 24 h oxaliplatin incubation (30 μM), total intracellular Pt (Fig. 2h and Additional file 5: Figure S2C) and DNA-bound Pt (Fig. 2i and Additional file 5: Figure S2D) was markedly higher in lenti-miR-128-3p transfected cells than control cells, confirming that reduced cellular Pt content is an important mechanism of oxaliplatin resistance. After 24 h of oxaliplatin treatment, nuclear foci of γ-H_2_AX levels in lenti-miR-128-3p cells were significantly increased, but remained low in lenti-NC cells (Fig. 2j and Additional file 5: Figure S2E). Finally, to determine whether miR-128-3p sensitizes CRC cells to chemotherapeutic agents in vivo, lenti-miR-128-3p transfected HCT116OxR cells were implanted subcutaneously into nude mice then treated with oxaliplatin. Our data indicated that miR-128-3p overexpression significantly decreased oxaliplatin resistance in HCT116OxR xenografts in vivo (Fig. 2k and l). These data support our in vitro findings, indicating that miR-128-3p ameliorates oxaliplatin-resistant CRC in vitro and in vivo. Collectively, these results demonstrate that decreased miR-128-3p expression is indispensable for oxaliplatin resistance in CRC cells.

**Fig. 2:** miR-128-3p expression in CRC cell lines and its effect on oxaliplatin resistance. **a** RT-qPCR assay was performed to detect the miR-128-3p expression in parent and resistant CRC cells. **b** RT-qPCR assay was performed to detect the miR-128-3p expression in HCT116OxR cells transfected with lenti-miR-128-3p (Lv-128) and lenti-negative control (Ctrl). **c** CCK8 assay of HCT116OxR cells transfected with Lv-128 and Ctrl with oxaliplatin treatment at indicated concentrations. **d** Flow cytometry for apoptosis assay of HCT116OxR cells transfected with Lv-128 and Ctrl with oxaliplatin treatment (30 μM). **e** Western blot analysis of E-cad, N-cad, Vim, and Fn expression in HCT116OxR cells transfected with Lv-128 and Ctrl. **f** Migration and invasion ability of HCT116OxR cells transfected with Lv-128 and Ctrl were assessed by Transwell assay. **g** Motility ability of HCT116OxR cells transfected with Lv-128 and Ctrl were assessed by wound healing assays. **h** Accumulation of Pt in HCT116OxR cells transfected with Lv-128 and Ctrl following exposure to 30 μM, 24 h oxaliplatin treatment. **i** Total Pt-DNA adduct levels in HCT116OxR cells transfected with Lv-128 and Ctrl following exposure to 30 μM, 24 h oxaliplatin treatment. **j** The immunofluorescence analysis of nuclear foci for γ-H_2_AX expression in HCT116OxR cells transfected with Lv-128 or Ctrl after 24 h oxaliplatin exposure (30 μM). Scale bars, 10 μm. Subcutaneous xenograft assay of miR-128-3p-overexpressing and control HCT116OxR cells (5 × 10^6^ cells) in nude mice with vehicle (veh) or oxaliplatin (Oxa, 90 mg/m^2^) treatment. Tumor volume of xenograft models were measured from day 0 to day 42. Volumes of tumors (k) and representative bioluminescent images (l) are shown (*n* = 5). Results are presented as mean ± SD. *P < 0.05, **P < 0.01, ***P < 0.001

### miR-128-3p levels in tumor tissues correlate with oxaliplatin response in CRC patients

As we observed miR-128-3p was substantially downregulated in both HCT116OxR and HT29OxR cells compared to parental cells, we felt it was important to establish clinical relevance in human CRC. Therefore, we analyzed miR-128-3p tissue levels in an independent large-scale sample set using RT-qPCR. Kruskal–Wallis test analysis indicated miR-128-3p expression levels in tissues were significantly lower in patients suffering from tumor relapse after oxaliplatin therapy (0.065; 0.033–0.088) compared with patients that responded well to neoadjuvant oxaliplatin therapy (0.169; 0.101–0.237) or who were therapy naive (0.204; 0.086–0.277) (all at *P* < 0.001). Compared with noncancerous tissues (1.014; 0.937–1.904), miR-128-3p expression levels were also markedly reduced in CRC tissues (*P* < 0.001, Fig. 3a and Additional file 1: Figure Table S1). We then explored the predictive value of miR-128-3p levels for oxaliplatin response in CRC patients. Expression levels of miR-128-3p were downregulated in patients with progressive disease (PD) during oxaliplatin therapy than those without PD (non-PD) (Fig. 3b). Receiver operating characteristic (ROC) curve analyses showed that miR-128-3p has a strong capability for discriminating non-PD patients from PD patients with an area under ROC curve (AUC) value of 0.868 (95% CI: 0.770–0.935, Fig. 3c). At an optimal cut-off value of 0.227, the sensitivity and specificity were 65.0 and 91.4%. Furthermore, the median miR-128-3p expression level (0.269) was used to categorize CRC patients into two groups; high-level (*n* = 61) and low-level (*n* = 61). Similar clinical characteristics between control and oxaliplatin treatment groups were observed before treatment. Associations between miR-128-3p and pathologies of CRC patients in validation phase are summarized in Additional file 2: Figure Table S3. Although Kaplan–Meier survival analysis indicated higher miR-128-3p expression was associated with longer progression-free survival (PFS) in CRC patients, there is limited benefit (Fig. 3d). Patients with low miR-128-3p expression had a poor PFS in oxaliplatin treatment (Fig. 3e). Conversely, the high miR-128-3p expression group exhibited a superior PFS after receiving oxaliplatin compared to the control group (Fig. 3f). Cox regression univariate and multivariate analysis revealed that oxaliplatin therapy correlated with improved PFS of CRC patients with high miR-128-3p expression (Table 1). Thus, miR-128-3p could serve as an independent predictor for oxaliplatin response in CRC patients.

**Fig. 3:** Expression level of miR-128-3p is correlate with oxaliplatin treatment response in CRC patients. **a** RT-qPCR analysis of miR-128-3p in CRC tissues from healthy donors (HD, *n* = 20) and patients who were therapy naive (Untreated, *n* = 18), benefited from neoadjuvant oxaliplatin therapy (Neoadjuvant, *n* = 18) and relapsed during oxaliplatin therapy (Post-relapse, *n* = 15). **b** RT-qPCR analysis of miR-128-3p in the pre-therapy tissue of CRC patients with non-PD (*n* = 35) or PD (*n* = 40) during oxaliplatin therapy. **c** ROC curves for detection of oxaliplatin using miR-128-3p as assessed by AUC. Kaplan–Meier survival curves analysis of PFS in CRC patients with or without oxaliplatin therapy. **d** All patients (*n* = 122); e. Patients with low miR-128-3p expression (*n* = 61); f. Patients with high miR-128-3p expression (*n* = 61). The median value of miR-128-3p expression level was used as a cut-off. Results are presented as mean ± SD. *P < 0.05, **P < 0.01, ***P < 0.001

**Table 1:** Univariate and multivariate analysis of factors associated

Variables	Low miR-128 (*n* = 61)		High miR-128 (*n* = 61)	
	Harzard ratio (95% CI)	*P* value	Harzard ratio (95% CI)	*P* value
Univariate analysis				
Oxaliplatin vs control	0.734(0.405–1.330)	0.308	0.295(0.137–0.637)	0.002*
Gender (male vs female)	1.310(0.732–2.345)	0.363	1.190(0.559–2.534)	0.652
Age (> 60 vs ≤60 years)	1.197(0.670–2.141)	0.544	1.215(0.571–2.586)	0.613
Tumor size (≤4 vs > 4 cm)	1.411(0.781–2.550)	0.253	0.720(0.315–1.645)	0.436
Tumor location (Rectum vs colon)	0.618(0.340–1.121)	0.113	1.293(0.600–2.789)	0.512
Tumor differentiation (Well/Moderate vs Poor)	0.890(0.492–1.611)	0.701	0.802(0.372–1.729)	0.573
TNM stage (II vs III/IV)	0.559(0.280–1.118)	0.100	1.259(0.435–3.646)	0.671
Distant metastasis (NO vs YES)	1.117(0.587–2.124)	0.736	2.203(0.883–5.498)	0.090
Multivariate analysis				
Oxaliplain vs control			0.311(0.140–0.688)	0.004*
Gender (male vs female)			0.947(0.391–2.293)	0.905
Age (> 60 vs ≤60 years)			0.898(0.385–2.093)	0.803
Tumor size (≤4 vs > 4 cm)			0.805(0.285–2.276)	0.683
Tumor location (Rectum vs colon)			0.913(0.315–2.650)	0.868
Tumor differentiation (Well vs Moderate/Poor)			1.210(0.412–3.551)	0.729
TNM stage (II vs III/IV)			1.046(0.306–3.576)	0.943
Distant metastasis (NO vs YES)			2.014(0.484–8.380)	0.336

### miR-128-3p is highly expressed and secreted by miR-128-3p transfected FHC cells and can be transferred to resistant CRC cells via exosome secretion

Previous studies suggest miRNAs can be packaged into exosomes and functionally delivered to target cells to directly modulate target mRNAs [29]. Herein, we transfected FHC cells with lenti-miR-128-3p or lenti-NC. Subsequently, extracellular exosomes were isolated from the FHC supernatant after 48 h and identified with electron microscopy by their typical cup-shaped morphology (40 to 120 nm) and by exosomal markers (CD63 + CD9 + GM130-) (Fig. 4a and b). The miR-128-3p expression was markedly higher in lenti-miR-128-3p FHC cells (FHC-128) and their exosomes (128-exo) than in lenti-NC FHC (FHC-NC) and associated exosomes (NC-exo) (Additional file 5: Figure S2F and Fig. 4c). We then determined whether miR-128-3p was indeed present within exosomes. As expected, miR-128-3p expression in culture medium was unchanged upon RNase A treatment but significantly decreased when treated with RNase A and Triton X-100 simultaneously (Fig. 4d), suggesting that released miR-128-3p was protected by double-layer membrane instead of being directly released. When 128-exo (labeled with membrane phospholipid dye PKH67) were incubated with HCT116OxR cells, recipient cells exhibited high uptake efficiency, as measured by laser scanning confocal microscope (Fig. 4e). After 24 h` incubation, > 80% of recipient cells were positive for PKH67 fluorescence (Additional file 6: Figure S3A), suggesting that 128-exo are effectively internalized by HCT116OxR cells. 128-exo co-incubations increased miR-128-3p levels in resistant cells nearly 350-fold, while NC-exo did not affect miR-128-3p expression levels (Fig. 4f and Additional file 6: Figure S3B). Moreover, prolonged incubation caused a corresponding increase in miR-128-3p levels in HCT116OxR cells (Fig. 4g). Additionally, actinomycin D (RNA polymerase II inhibitor) did not significantly alter miR-128-3p levels, excluding the possibility of endogenous induction of miR-128-3p in recipient resistant cells (Fig. 4h). Taken together, these data demonstrate FHC-128 cells efficiently secrete exosomes containing miR-128-3p that can be directly transferred to HCT116OxR cells.

**Fig. 4:** Characterization and roles of exosomes derived from miR-128-3p transfected FHC cells. **a** Left: exosomes were analyzed under electron microscopy which displayed the same morphology. Scale bar = 200 nm. Right: Nanoparticle tracking analysis were analyzed the size distribution and number of exosomes derived from FHC cells. **b** Western blotting analysis showing exosome-enriched medium with expression of the exosome marker of CD63 and CD9 and non-expression of the cis-Golgi matrix protein (GM130). **c** RT-qPCR detection of miR-128-3p expression in exosome derived from FHC cells transfected with Lv-128 and Ctrl. **d** RT-qPCR analysis of miR-128-3p in the 128-exo cocultured cells were untreated with or treated with RNase A (10 μg/ml) and/or 0.3% Triton X-100 and then further mixed with of RNase inhibitor. **e** Internalization of exosome derived from FHC-128 cells. Labelled 128-exo (green fluorescent dye, PKH67) were uptake by HCT116OxR (DAPI-labelled) cells. **f** RT-qPCR analysis of miR-128-3p in recipient HCT116OxR cells that were treated with PBS, NC-exo, 128-exo, 128-exo with anti-control (anti-ctrl) and anti-miR-128-3p (anti-128). **g** RT-qPCR analysis of miR-128-3p in recipient HCT116OxR cells co-cultured with different incubation time of 128-exo. **h** RT-qPCR analysis of miR-128-3p in HCT116OxR cells treated with Actinomycin D (ActD) (1 μg/mL) followed by 128-exo treatment for 48 h. Results are presented as mean ± SD. *P < 0.05, **P < 0.01, ***P < 0.001

### Exosome-mediated transfer of miR-128-3p reversed oxaliplatin resistance through altering target gene expression

We next investigated whether exosome-transferred miR-128-3p could ameliorate chemosensitivity in resistant cells. In a cell viability and Annexin V/PI apoptosis assay, oxaliplatin-resistant cells incubated directly with 128-exo displayed elevated oxaliplatin sensitivity (Fig. 5a, b and Additional file 6: Figure S3C–E) which was abolished by transfecting recipient cells with a miR-128-3p inhibitor (anti-128). To exclude other factors in exosomes besides miR-128-3p in mediating oxaliplatin sensitivity, we electroporated miR-128-3p mimics directly into exosomes and it did not affect the physical properties of the exosomes (Additional file 6: Figure S3F). Indeed, HCT116OxR cells co-cultured with exosomes successfully up-took miR-128-3p mimics (Additional file 6: Figure S3G) and also exhibited increased oxaliplatin sensitivity (Additional file 6: Figure S3H). Importantly, incubated with 128-exo suppressed EMT, as characterized by upregulation of epithelial markers and downregulation of mesenchymal markers in resistant cells, while anti-128 blocked this progression (Fig. 5c and Additional file 7: Figure S4A–C). Moreover, 128-exo suppressed migration and invasion of resistant CRC cells across Transwell filters (Fig. 5d and Additional file 7: Figure S4D). And wound healing assays further showed that 128-exo suppressed motility in resistant cells (Fig. 5e and Additional file 7: Figure S4E). Both these affects were abolished with addition of anti-128. Using atomic absorption spectroscopy (AAS), we found that the total intracellular Pt and DNA-bound Pt levels in resistant cells was significantly increased when treated with 128-exo (Fig. 5f, g Additional file 7: Figure S4F, G). At 24 h` post oxaliplatin treatment, the nuclear foci of γ-H_2_AX levels in the control group remained low but were significantly increased in the 128-exo co-culture group (Fig. 5h and Additional file 8: Figure S5A). Additionally, we found that the restored oxaliplatin sensitivity in recipient cells was sustained for at least 10 days following removal of 128-exo (Additional file 8: Figure S5B). Importantly, intra-tumor injection of miR-128-3p exosomes restored oxaliplatin response in resistant cells in vivo (Fig. 5i and j) and was accompanied by an increase in tumor miR-128-3p levels (Additional file 8: Figure S5C). Furthermore, miR-128-3p mimic-loaded exosomes were also effective. Therefore, these results confirm that miR-128-3p overexpression through 128-exo reverses oxaliplatin resistance in CRC cells in vitro and vivo.

**Fig. 5:** Intercellular transfer of miR-128-3p by 128-Exo sensitizes CRC cells to oxaliplatin agents. **a** CCK8 assay of HCT116OxR cells pre-incubated with indicated factors for 48 h followed by oxaliplatin treatment at indicated concentrations. **b** Flow cytometry for apoptosis assay of HCT116OxR cells pre-incubated with indicated factors for 48 h followed by oxaliplatin treatment (30 μM) for 24 h. **c** Western blot analysis of protein E-cad, N-cad, Vim, and Fn expression in HCT116OxR cells after incubated with indicated factors. **d** Migration and invasion ability of HCT116OxR cells after incubated with indicated factors for 48 h were assessed by Transwell assays. **e** Motility ability of HCT116OxR cells after incubated with indicated factors for 48 h were assayed by wound healing assays. **f** Accumulation of Pt in HCT116OxR cells after incubated with indicated factors for 48 h following exposure to 30 μM, 24 h oxaliplatin treatment. **g** Total Pt-DNA adduct levels in HCT116OxR cells after incubated with indicated factors for 48 h following exposure to 30 μM, 24 h oxaliplatin treatment. **h** Immunofluorescence analysis of nuclear foci for γ-H_2_AX expression HCT116OxR cells incubated with indicated factors for 48 h followed by 24 h` oxaliplatin exposure (30 μM). Scale bars, 10 μm. **i** Subcutaneous xenograft assay of HCT116OxR cells (5 × 10^6^ cells) in nude mice with intratumoral injection of PBS, 128-exo and exo/FHC miR-128-3p electrop in nude mice with vehicle or oxaliplatin (90 mg/m^2^) treatment. Tumor volume of xenograft models were measured from day 0 to day 42. Volumes of tumors (i) and representative bioluminescent images (j) are shown (*n* = 5 per group). Results are presented as mean ± SD. *P < 0.05, **P < 0.01, ***P < 0.001.

### Bmi1 and MRP5 are responsible for miR-128-3p-mediated oxaliplatin resistance

We further sought to identify the mediators of miR-128-3p-driven oxaliplatin resistance. Previous reports suggest interactions of Bmi1/E-cadherin and ATP-dependent glutathione S-conjugate export pump (e.g. MRP5) are important regulators [30–32]. To identify the potential pathway, we performed bioinformatic analysis with TargetScan and Miranda. This revealed the 3`-UTR of Bmi1 and MRP5 contain a predicted binding site for miR-128-3p (Fig. 6a). Furthermore, we found an inverse correlation between miR-128-3p levels and Bmi1 mRNA (r = − 0.445, *P* < 0.001) or MRP5 expression mRNA (r = − 0.538, *P* < 0.001) in CRC tissues (Fig. 6b and c). To verify whether Bmi1 and MRP5 are direct targets of miR-128-3p, Dual-Luciferase reporter system with pmiR-REPORT™ luciferase vectors containing wild-type or mutant 3`-UTR of Bmi1 and MRP5 was used. Co-transfection of miR-128-3p mimics significantly suppressed the luciferase activity of the reporter containing wild-type 3`-UTR, but not the mutant reporter (Additional file 9: Figure S6A and B). These data reveal that Bmi1 and MRP5 are direct functional targets of miR-128-3p. RT-qPCR and western blot assay indicated that the Bmi1 and MRP5 mRNA and protein levels were lower in miR-128-3p overexpressing cells compared to controls (Additional file 9: Figure S6C–E). To further validate these results, we employed a ‘rescue’ experiment by transfecting pcDNA3.1 vector carrying Bmi1 or MRP5 expression cassette with wild or mutated type seed sequences for miR-128-3p (Bmi-wt/Bmi1-mut or MRP5-wt/MRP5-mut) at its 3`-UTR into lenti-miR-128-3p transfected resistant cells. A cell viability and apoptosis assay indicated that only transfection of resistant cells with Bmi1-mut or MRP5-mut developed a resistant phenotype, while co-transfection with a Bmi1-wt or MRP5-wt did not and were silenced by miR-128-3p (Fig. 6d, e and Additional file 9: Figure S6F–H). Western blots assay demonstrated that transfecting resistant cells with Bmi1-mut permitted Bmi1, N-cadherin, vimentin, and fibronectin protein expression and suppressed E-cadherin protein expression, while transfection with Bmi1-wt was silenced by miR-128-3p and could not recover EMT (Fig. 6f and Additional file 10: Figure S7A). Moreover, ‘rescuing’ Bmi1-mut expression in the presence of miR-128-3p enhanced the invasion and migration of HCT116OxR cells (Fig. 6g, h and Additional file 10: Figure S7B, C). Collectively, these data suggest that miR-128-3p regulates chemotherapy-induced EMT of CRC cells by targeting Bmi1. We further sought to identify the drug efflux mechanism of miR-128-3p-driven oxaliplatin resistance. Western blotting revealed a significant increase in MRP5 protein in the MRP5-mut transfected cells, as MRP5 proteins in the mock, control groups or cells transfected with MRP5-wt remained unchanged (Fig. 6i and Additional file 10: Figure S7D). Importantly, transfected MRP5-mut significantly decreased the total intracellular Pt and DNA-bound Pt in lenti-miR-128-3p transfected HCT116OxR cells compared with the cells transfected with mock, control and MRP5-wt (Fig. 6j, k and Additional file 10: Figure S7E, F). The nuclear foci of γ-H_2_AX expression levels revealed that oxaliplatin induced less DNA damage at 24 h in MRP5-mut group than other groups in lenti-miR-128-3p transfected resistant cell lines (Fig. 6l and Additional file 10: Figure S7G). In addition, treatment with 128-exo significantly decreased Bmi1 and MRP5 expression at protein levels in resistant cell lines, and miR-128-3p inhibitor in recipient cells disrupted this effect (Fig. 6m and Additional file 10: Figure S7H). Furthermore, forced miR-128-3p expression through intra-tumor injection of exosomes restored oxaliplatin response in resistant cells through blocked Bmi1 and MRP5 associated signaling in vivo (Fig. 6n). These findings indicate that 128-exo potentially facilitates oxaliplatin sensitivity in CRC cells by negatively regulating Bmi1 and MRP5 expression, two genes involved in oxaliplatin-induced EMT and drug efflux respectively.

**Fig. 6:** Exosomes containing miR-128-3p sensitized CRC cells to oxaliplatin by targeting to Bmi1 and MRP5. **a** Illustration of the putative predicted miR-128-3p binding site in the Bmi1 and MRP5 mRNA 3`-UTR region. **b** Spearman’s correlation analysis between Bmi1 mRNA levels and miR-128-3p levels in CRC tissues. **c** Spearman’s correlation analysis between MRP5 mRNA levels and miR-128-3p levels in CRC tissues. **d** CCK8 assay of Lv-128 transfected HCT116OxR cells in different conditions followed by oxaliplatin treatment at indicated concentrations. **e** Flow cytometry for apoptosis assay of Lv-128 transfected HCT116OxR cells in different conditions followed by oxaliplatin treatment (30 μM) for 24 h. **f** Western blot analysis of protein Bmi1, E-cad, N-cad, Vim, and Fn expression of Lv-128 transfected HCT116OxR cells in different conditions. **g** Migration and invasion ability of Lv-128 transfected HCT116OxR cells in different conditions were assessed by Transwell assays. **h** Motility ability of Lv-128 transfected HCT116OxR cells in different conditions were assayed by wound healing assays. **i** Western blot analysis of protein MRP5 expression of Lv-128 transfected HCT116OxR cells in different conditions. **j** Accumulation of Pt in Lv-128 transfected HCT116OxR cells in different conditions following exposure to 30 μM, 24 h oxaliplatin treatment. **k** Total Pt-DNA adduct levels in Lv-128 transfected HCT116OxR cells in different conditions following exposure to 30 μM, 24 h oxaliplatin treatment. **l** Immunofluorescence analysis of nuclear foci for γ-H_2_AX expression of Lv-128 transfected HCT116OxR cells in different conditions after 24 h oxaliplatin exposure (30 μM). Scale bars, 10 μm. **m** Western blot analysis of protein Bmi1 and MRP5 expression in HCT116OxR cells after incubated with indicated factors. **n** Immunohistochemistry analysis of Bmi1 and MRP5 protein levels in xenograft tumor tissues with intratumoral injection of NC-exo and 128-exo (20×). Results are presented as mean ± SD. *P < 0.05, **P < 0.01, ***P < 0.001

## Discussion

Presently, advanced CRC patients who develop oxaliplatin resistance have limited therapeutic options. Hence, it is necessary to investigate the biological basis of oxaliplatin resistance and identify novel therapeutic targets and prevention strategies for oxaliplatin resistance. This study identified miR-128-3p as an important antitumor microRNA and inhibitor of tumor progression. miR-128-3p is downregulated in oxaliplatin-resistant CRC and functionally required to the suppress the drug resistant phenotype. miR-128-3p overexpression re-sensitizes oxaliplatin response by competitively binding Bmi1 and MRP5 mRNA 3`-UTR, leading to the mesenchymal-epithelial transition of oxaliplatin-resistant CRC cells and reduced cellular oxaliplatin efflux. We also demonstrated a novel strategy to increase CRC chemosensitivity using exosomes to transfer therapeutic miR-128-3p into resistant CRC cells. The miR-128-3p modified FHC cells effectively packages miR-128-3p into secreted exosomes, and mediates miR-128-3p transfer to oxaliplatin-resistant CRC cells. Consequently rendering resistant CRC cells more sensitive to chemotherapeutic agents by altering Bmi1 and MRP5 expression (Fig. 7).

**Fig. 7:** A schematic diagram of exosomal miR-128-3p based signaling pathway in CRC treatment. In oxaliplatin-resistant CRC cells, exosomal miR-128-3p derived from FHC-128 cells reverse oxaliplatin resistance by competitively binding Bmi1 and MRP5, leading to the increased expression of E-cadherin (suppress EMT phenotype) and reduced the oxaliplatin efflux

Mir-128 has been described as a tumor suppressor, and a reduced level of miR-128 was first identified in glioblastoma [33]. Recent studies suggested that aberrant miR-128-3p expression has been observed in some malignant cancer cell phenotypes such as: self-renewal, proliferation, apoptosis, cell motility, and invasion [11, 34, 35]. Here, we extend the current knowledge by highlighting the role of miR-128-3p in chemotherapy-resistant CRC. Our results demonstrated that miR-128-3p expression levels in CRC tumor tissues and cell lines were significantly lower than normal tissues and cell lines. Additionally, downregulated miR-128-3p was identified in oxaliplatin-resistant cells compared with sensitive cells. Therefore, we speculate that miR-128-3p might play important roles in oxaliplatin-resistant CRC.

Understanding the mechanisms of drug resistance in CRC is essential for optimizing current therapeutic strategies. We explored the potential mechanisms underlying miR-128-3p mediated reversal of chemoresistance by focusing on likely molecular targets. Here, we identified polycomb group protein Bmi1 as a functional target of miR-128-3p to regulate EMT. Previous studies have shown that downregulation of Bmi1 could restrain cell proliferation, arrest cell cycle, promote cell apoptosis, and inhibit cell self-renewal which is essential for CRC initiating cells [36]. In our previous study, Bmi1 is highly expressed in CRC and is a potential biomarker for diagnosis and prognosis [37]. Consistent with the observations that Bmi1 is essential in Twist1-induced epithelial–mesenchymal transition through repressed expression of E-cadherin in head and neck squamous cell carcinoma [30], our study found that miR-128-3p positively regulated E-cadherin expression in CRC cells through binding the Bmi1 3`-UTR. Therefore, Bmi1 overexpression due to reduced miR-128-3p may result in chemotherapy-induced EMT in CRC via this pathway. Additionally, we found that MRP5 (also known as ABCC5), a member of the ABC transporter family, was also a target of miR-128-3p. The human ABC genes encode ATP-dependent transporters that can move substrates, against their electrochemical gradient, in both directions across biological membranes (cell and vesicles) [38]. Accumulating evidence suggests that increased MRP5 expression is associated with exposure to platinum drugs in lung cancer in vivo and/or the chronic stress response to xenobiotics [39]. Increased resistance to platinum drugs with elevated MRP5 levels may be due to glutathione S-platinum complex efflux. Our findings provide evidence that highly expressed miR-128-3p reduce oxaliplatin export by down-regulating MRP5 expression in cancer cells. Moreover, decreased oxaliplatin efflux could result in higher tissue distribution and intracellular drug localization to form damaging DNA-platinum adducts that ultimately destroy tumor cells. In short, our results demonstrate that compared with parent cells, miR-128-3p expression was significantly downregulated in oxaliplatin-resistant cells. Overexpression of miR-128-3p could reestablish sensitivity in resistant cells by reducing Bmi1 and MRP5 expression which related to oxaliplatin-resistance. Oxaliplatin combined with miR-128-3p overexpression inhibited the development of resistant CRC cells more effectively than oxaliplatin alone in vitro and in vivo.

Oxaliplatin therapy might have unrealized clinical benefits in the selection of oxaliplatin-responsive CRC patients that are masked due to a lack of biomarkers. Therefore, the identification of reliable predictive biomarkers for clinical benefits of oxaliplatin therapy is urgently needed. Ideal biomarkers, like microRNAs, are advantageous because they are more stable than other biological macromolecules. Herein, we performed the first investigation into the prognostic value of miR-128-3p for CRC oxaliplatin-resistance. Our results showed that lower miR-128-3p expression in pre-therapy CRC tumors significantly correlates with a poor oxaliplatin response. Moreover, our results demonstrated that miR-128-3p effectively distinguished resistant patients from sensitive patients, with a significantly higher AUC value of 0.868, as well as a sensitivity of 65.0% and specificity of 91.4% at optimal cut-off value of 0.227. We also estimated the prognostic power of miR-128-3p through Kaplan-Meier survival analysis. Patients with high miR-128-3p expression exhibited dramatic improved prognosis following oxaliplatin treatment. Taking this further, univariate and multivariate Cox model analyses showed that miR-128-3p was an independent prognostic factor. Therefore, when determining a course of treatment, we advise evaluating miR-128-3p expression in CRC tumors to predict patients who might benefit from oxaliplatin therapy. In treatment-naive patients with low miR-128-3p levels, we suggest therapeutic to increase miR-128-3p expression as we found this enhances response to oxaliplatin.

It is very important to contrast exogenous synthetic siRNAs with microRNAs which are endogenous molecules in normal cells with potentially fewer unexpected off-target silencing effects [40, 41]. Since a microRNA molecule targets a set of coding genes, rather than a single one, therapies based on microRNA interference could be more potent in cancer treatment by targeting multiple molecular pathways. Exosomes have the capacity to protect cellular contents like miRNAs [42] from degradation in circulation and function as carriers to transmit their donor cells’ contents to recipient cells [43]. Although liposomes may also offer advantages for therapeutic molecule delivery over viral-based delivery systems, they exhibit low efficiency and rapid clearance from the circulation [44]. Unlike liposomes, exosomes contain membrane anchored and transmembrane proteins that functionally enhance endocytosis, thus promoting the delivery of their internal content [45, 46]. Exosomal proteins, such as CD47, allows for evasion from phagocytosis by the circulating monocytes and increases exosomes half-life in the circulation [47, 48]. Moreover, recent evidence suggest that exosomes exhibit a superior ability to deliver “drugs” and suppress tumor growth when compared to liposomes [49]. In addition, using exosomes might also minimize cytotoxic effects when synthetic nanoparticles were used in vivo [50]. Meanwhile, because of their nanosize, exosomes are explored as nanodevices for the development of new therapeutic applications. Mesenchymal stem cell-derived exosomes containing the prodrug 5-fluorocytosine (5-FC) were internalized by recipient tumor cells. The endocytosed exosomes effectively triggered a dose-dependent tumor cell death following the intracellular conversion of the prodrug 5-FC to 5-fluorouracil [51]. Hence, natural exosomes are of considerable interest because they can be used as biological delivery vehicles for targeted tumor therapy [52, 53]. In this study, we demonstrated a novel strategy for increasing CRC chemosensitivity through 128-exo mediated transfer of therapeutic miR-128-3p. Our work shows that exosomes derived from miR-128-3p overexpressing FHC can deliver miR-128-3p into oxaliplatin-resistant CRC cells in vitro and in vivo, further restoring CRC cell sensitivity to chemotherapeutic agents by altering the expression of target genes Bmi1 and MRP5 in resistant cells. Therefore, by decreasing the expression of target genes, exosomes from miR-128-3p-modified FHCs can effectively increase the chemo-sensitivity of CRC cells through the suppression of EMT and drug efflux. Given that systemic therapy with oxaliplatin is the standard of care for advanced-stage CRC [54], we further tested whether 128-exo can exert its inhibitory function in a mouse model. A lower concentration of oxaliplatin (90 mg/m^2^) than the clinical amount was used to treat CRC xenograft tumors. Immunohistochemistry assay results demonstrated that intra-tumor injection of 128-exo significantly enhanced the tumor suppression at lower oxaliplatin concentrations through decreased expression of Bmi1 and MRP5. Additionally, in vitro experiments indicated 128-exo treatment reduced gene expression in CRC cells over time, up to ten days after 128-exo treatment.

## Conclusion

Our findings demonstrate that miR-128-3p acts not only as a clinical biomarker for oxaliplatin response but also as a therapeutic target. miR-128-3p delivery via exosomes increases the sensitivity of CRC cells to oxaliplatin, thereby providing a new treatment strategy for CRC.

## Additional files

Additional file 1: **Table S1.** Clinical characteristics of CRC patients in training phase. (DOCX 19 kb)

Additional file 2: **Table S3.** Clinical characteristics of 122 CRC patients in indicated groups. (DOCX 16 kb)

Additional file 3: **Table S2.** Primer sequence and antibody. (DOCX 18 kb)

Additional file 4: **Figure S1.** related to Fig. 2. miR-128-3p expression in CRC cell lines and its effect on oxaliplatin resistance. A. CCK8 assay of seven CRC cell lines (LoVo, HT29, SW480, SW620, HCT116, SW1116 and Caco2) followed by oxaliplatin treatment at indicated concentrations. B. A representative scatter-gram of Annexin V/PI potential test for parent and resistant cell apoptosis. C. RT-qPCR assay was performed to detect the miR-128-3p expression in seven CRC cell lines (LoVo, HT29, SW480, SW620, HCT116, SW1116 and Caco2) and normal FHC cells. D. RT-qPCR assay was performed to detect miR-128-3p expression in HT29OxR cells transfected with lenti-miR-128-3p (Lv-128) and lenti-negative control (Ctrl). E. CCK8 assay of HT29OxR cells transfected with Lv-128 and Ctrl with oxaliplatin treatment at indicated concentrations. F. Flow cytometry apoptosis assay of HT29OxR cells transfected with Lv-128 and Ctrl with oxaliplatin treatment (30 μM) for 24 h. G. A representative scatter-gram of Annexin V/PI potential test for HCT116OxR (upper) and HT29OxR (lower) cell apoptosis. H. RT-qPCR analysis of E-cadherin (E-cad), N-cadherin (N-cad), vimentin (Vim), and fibronectin (Fn) expression in HCT116OxR cells transfected with Lv-128 and Ctrl. I. RT-qPCR analysis of E-cad, N-cad, Vim, and Fn expression in HT29OxR cells transfected with Lv-128 and Ctrl. J. Western blot analysis of E-cad, N-cad, Vim, and Fn expression in HT29OxR cells transfected with Lv-128 and Ctrl. (TIF 1091 kb)

Additional file 5: **Figure S2.** related to Fig. 2. miR-128-3p expression in CRC cell lines and its effect on oxaliplatin resistance. A. Migration and invasion ability of HT29OxR cells transfected with Lv-128 and Ctrl were assessed with a Transwell assay. B. Motility ability of HT29OxR cells transfected with Lv-128 and Ctrl were assessed by wound healing assays. C. Accumulation of Pt in HT29OxR cells transfected with Lv-128 or Ctrl following exposure to 30 μM oxaliplatin treatment for 24 h. D. Total Pt-DNA adduct levels in HT29OxR cells transfected with Lv-128 or Ctrl following exposure to 30 μM oxaliplatin treatment for 24 h. E. The immunofluorescence analysis of nuclear foci for γ-H_2_AX expression induced by oxaliplatin in HT29OxR cells transfected with Lv-128 or Ctrl after 24 h` oxaliplatin exposure (30 μM). Scale bars, 10 μm. F. RT-qPCR assay was performed to detect the miR-128-3p expression in FHC cells transfected with Lv-128 or Ctrl. (TIF 1535 kb)

Additional file 6: **Figure S3.** related to Fig. 5. Intercellular transfer of miR-128-3p by 128-Exo sensitized CRC cells to oxaliplatin agents. A. Internalization of exosomes derived from FHC-128 cells. Labelled 128-exo (green fluorescent dye, PKH67) were uptake by HCT116OxR (DAPI-labelled) cells. B. RT-qPCR analysis of miR-128-3p in HT29OxR cells pre-incubated with indicated factors. C. CCK8 assay of HT29OxR cells pre-incubated with indicated factors for 48 h followed by oxaliplatin treatment at indicated concentrations. D. Flow cytometry apoptosis assay of HT29OxR cells pre-incubated with indicated factors for 48 h followed by oxaliplatin treatment (30 μM) for 24 h. E. A representative scatter-gram of Annexin V/PI potential test for HCT116OxR (upper) and HT29OxR (lower) cell apoptosis. F. Exosomes were imaged using electron microscopy. Scale bar = 200 nm. G. RT-qPCR assay was performed to detect miR-128-3p expression in HCT116OxR cells following various treatments. H. CCK8 assay of HCT116OxR cells pre-incubated with indicated factors for 48 h followed by oxaliplatin treatment at indicated concentrations. (TIF 1395 kb)

Additional file 7: **Figure S4.** related to Fig. 5. Intercellular transfer of miR-128-3p by 128-Exo sensitized CRC cells to oxaliplatin agents. A. RT-qPCR analysis of E-cad, N-cad, Vim, and Fn mRNA expression in HCT116OxR cells after incubated with indicated factors for 48 h. B. RT-qPCR analysis of E-cad, N-cad, Vim, and Fn mRNA expression in HT29OxR cells after incubated with indicated factors for 48 h. C. Western blot analysis of protein E-cad, N-cad, Vim, and Fn expression in HT29OxR cells after incubated with indicated factors for 48 h. D. Migration and invasion ability of HT29OxR cells after incubated with indicated factors for 48 h were assessed by Transwell assays. E. Motility ability of HT29OxR cells after incubated with indicated factors for 48 h were assayed by wound healing assays. F. Accumulation of Pt in HT29OxR cells after incubated with indicated factors for 48 h followed by exposure to 30 μM, 24 h oxaliplatin treatment. F. Total Pt-DNA adduct levels in HT29OxR cells after incubated with indicated factors for 48 h following exposure to 30 μM, 24 h oxaliplatin treatment. (TIF 1549 kb)

Additional file 8: **Figure S5.** related to Fig. 5. Intercellular transfer of miR-128-3p by 128-Exo sensitized CRC cells to oxaliplatin agents. A. The immunofluorescence analysis of nuclear foci for γ-H_2_AX expression in HT29OxR cells after incubated with indicated factors for 48 h followed by 24 h oxaliplatin exposure (30 μM). B. HCT116OxR cells were incubated with PBS, NC-exo and 128-exo for 48 h and replaced with fresh culture medium. The oxaliplatin IC50 at subsequent 0 day, 5 day and 10 day were determined by CCK8 assay. C. RT-qPCR analysis of miR-128-3p expression in xenograft tissues after incubated with indicated factors. (TIF 602 kb)

Additional file 9: **Figure S6.** related to Fig. 6. Exosomes containing miR-128-3p sensitized CRC cells to oxaliplatin by targeting to Bmi1 and MRP5. Luciferase activity assay was performed for the cells co-transfected with pmiR-REPORT™ vectors containing Bmi1-wt 3`-UTR/Bmi1-mut 3`-UTR sequences (A) or MRP5-wt 3`-UTR/MRP5-mut 3`-UTR sequences (B) and miR-128-3p mimics. Data are presented as normalized fold change in luciferase activity. RT-qPCR assay was performed to detect the Bmi1 mRNA (C) and MRP5 mRNA (D) expression in resistant cells transfected with Lv-128 and Ctrl. E. Western blot analysis of Bmi1 and MRP5 protein expression of HCT116OxR and HT29OxR cells transfected with Lv-128 and Ctrl. F. CCK8 assay of Lv-128 transfected HT29OxR cells treated with indicated factors for 48 h followed by oxaliplatin treatment at indicated concentrations. G. Flow cytometry for apoptosis assay of Lv-128 transfected HT29OxR cells treated with indicated factors for 48 h followed by oxaliplatin treatment (30 μM) for 24 h. H. A representative scatter-gram of Annexin V/PI potential test for HCT116OxR (upper) and HT29OxR (lower) cell apoptosis. (TIF 1078 kb)

Additional file 10: **Figure S7.** related to Fig. 6. Exosomes containing miR-128-3p sensitized CRC cells to oxaliplatin by targeting to Bmi1 and MRP5. A. Western blot analysis of Bmi1 and E-cad, N-cad, Vim, and Fn protein expression of Lv-128 transfected HT29OxR cells in different conditions. B. Migration and invasion ability of Lv-128 transfected HT29OxR cells in different conditions were assessed by Transwell assays. C. Motility ability of Lv-128 transfected HT29OxR cells in different conditions were assayed by wound healing assays. D. Western blot analysis of protein MRP5 expression of Lv-128 transfected HT29OxR cells in different conditions. E. Accumulation of Pt in lenti-miR-128-3p transfected HT29OxR cells in different conditions following exposure to oxaliplatin treatment 30 μM for 24 h. F. Total Pt-DNA adduct levels in Lv-128 transfected HT29OxR cells in different conditions following exposure to 30 μM, 24 h oxaliplatin treatment. G. Western blot analysis of γ-H_2_AX expression in Lv-128 transfected HT29OxR cells in different conditions 24 h after oxaliplatin exposure (30 μM). H. Western blot analysis of Bmi1 and MRP5 protein expression in HT29OxR cells after incubation with indicated factors. (TIF 1843 kb)

## Abbreviations

128-exo: Lenti-miR-128-3p transfected FHC cells derived exosomes
AAS: Atomic absorption spectrophotometry
AUC: Area under the receiver-operating characteristic curve
Bmi1: B-cell-specific moloney murine leukemia virus integration site 1
CRC: Colorectal cancer
FHC-128: Lenti-miR-128-3p transfected FHC cells
FHC-NC: Lenti-NC transfected FHC cells
IHC: Immunohistochemistry
lv-128: Lentiviral vector miR-128-3p
lv-NC: Lentiviral vector negative control
MRP5: Multidrug resistant protein 5
NC-exo: Lenti-NC transfected FHC cells derived exosomes
NTA: Nanoparticle tracking analysis
PFS: Progression-free survival
ROC: Receiver operating characteristic
RT-qPCR: Quantitive real-time polymerase chain reaction
TEM: Transmission electron microscopy
TNM: Tumor-node metastasis

## References

[1] Jemal A, Bray F, Center MM, Ferlay J, Ward E, Forman D (2011). Global cancer statistics. CA Cancer J Clin.

[2] Yang AD, Fan F, Camp ER, van Buren G, Liu W, Somcio R, Gray MJ, Cheng H, Hoff PM, Ellis LM (2006). Chronic oxaliplatin resistance induces epithelial-to-mesenchymal transition in colorectal cancer cell lines. Clin Cancer Res.

[3] Arango D, Wilson AJ, Shi Q, Corner GA, Aranes MJ, Nicholas C, Lesser M, Mariadason JM, Augenlicht LH (2004). Molecular mechanisms of action and prediction of response to oxaliplatin in colorectal cancer cells. Br J Cancer.

[4] Meads MB, Gatenby RA, Dalton WS (2009). Environment-mediated drug resistance: a major contributor to minimal residual disease. Nat Rev Cancer.

[5] Li H, Yang BB (2013). Friend or foe: the role of microRNA in chemotherapy resistance. Acta Pharmacol Sin.

[6] Holzel M, Bovier A, Tuting T (2013). Plasticity of tumour and immune cells: a source of heterogeneity and a cause for therapy resistance?. Nat Rev Cancer.

[7] McMillin DW, Negri JM, Mitsiades CS (2013). The role of tumour-stromal interactions in modifying drug response: challenges and opportunities. Nat Rev Drug Discov.

[8] Breunig C, Erdem N, Bott A, Greiwe JF, Reinz E, Bernhardt S, Giacomelli C, Wachter A, Kanthelhardt EJ, Beissbarth T (2018). TGFbeta1 regulates HGF-induced cell migration and hepatocyte growth factor receptor MET expression via C-ets-1 and miR-128-3p in basal-like breast cancer. Mol Oncol.

[9] Ambs S, Prueitt RL, Yi M, Hudson RS, Howe TM, Petrocca F, Wallace TA, Liu CG, Volinia S, Calin GA (2008). Genomic profiling of microRNA and messenger RNA reveals deregulated microRNA expression in prostate cancer. Cancer Res.

[10] Khan AP, Poisson LM, Bhat VB, Fermin D, Zhao R, Kalyana-Sundaram S, Michailidis G, Nesvizhskii AI, Omenn GS, Chinnaiyan AM, Sreekumar A (2010). Quantitative proteomic profiling of prostate cancer reveals a role for miR-128 in prostate cancer. Mol Cell Proteomics.

[11] Cai J, Fang L, Huang Y, Li R, Xu X, Hu Z, Zhang L, Yang Y, Zhu X, Zhang H (2017). Simultaneous overactivation of Wnt/beta-catenin and TGFbeta signalling by miR-128-3p confers chemoresistance-associated metastasis in NSCLC. Nat Commun.

[12] Xiao M, Lou C, Xiao H, Yang Y, Cai X, Li C, Jia S, Huang Y (2018). MiR-128 regulation of glucose metabolism and cell proliferation in triple-negative breast cancer. Br J Surg.

[13] Shan ZN, Tian R, Zhang M, Gui ZH, Wu J, Ding M, Zhou XF, He J (2016). miR128-1 inhibits the growth of glioblastoma multiforme and glioma stem-like cells via targeting BMI1 and E2F3. Oncotarget..

[14] Liu HT, Wang YW, Xing AY, Shi DB, Zhang H, Guo XY, Xu J, Gao P (2017). Prognostic value of microRNA signature in patients with gastric cancers. Sci Rep.

[15] Lian B, Yang D, Liu Y, Shi G, Li J, Yan X, Jin K, Liu X, Zhao J, Shang W (2018). Zhang R: miR-128 targets the SIRT1/ROS/DR5 pathway to sensitize colorectal Cancer to TRAIL-induced apoptosis. Cell Physiol Biochem.

[16] Sun Z, Shi K, Yang S, Liu J, Zhou Q, Wang G, Song J, Li Z, Zhang Z, Yuan W (2018). Effect of exosomal miRNA on cancer biology and clinical applications. Mol Cancer.

[17] Gonzalez-Begne M, Lu B, Han X, Hagen FK, Hand AR, Melvin JE, Yates JR (2009). Proteomic analysis of human parotid gland exosomes by multidimensional protein identification technology (MudPIT). J Proteome Res.

[18] Cheshomi H, Matin MM. Exosomes and their importance in metastasis, diagnosis, and therapy of colorectal cancer. J Cell Biochem. 2018. 10.1002/jcb.27582.10.1002/jcb.2758230246315

[19] Hu G, Drescher KM, Chen XM (2012). Exosomal miRNAs: biological properties and therapeutic potential. Front Genet.

[20] Katakowski M, Buller B, Zheng X, Lu Y, Rogers T, Osobamiro O, Shu W, Jiang F, Chopp M (2013). Exosomes from marrow stromal cells expressing miR-146b inhibit glioma growth. Cancer Lett.

[21] Li P, Zhang X, Wang H, Wang L, Liu T, Du L, Yang Y, Wang C (2017). MALAT1 is associated with poor response to Oxaliplatin-based chemotherapy in colorectal Cancer patients and promotes Chemoresistance through EZH2. Mol Cancer Ther.

[22] Qu L, Ding J, Chen C, Wu ZJ, Liu B, Gao Y, Chen W, Liu F, Sun W, Li XF (2016). Exosome-transmitted lncARSR promotes Sunitinib resistance in renal Cancer by acting as a competing endogenous RNA. Cancer Cell.

[23] Eisenhauer EA, Therasse P, Bogaerts J, Schwartz LH, Sargent D, Ford R, Dancey J, Arbuck S, Gwyther S, Mooney M (2009). New response evaluation criteria in solid tumours: revised RECIST guideline (version 1.1). Eur J Cancer.

[24] Thery C, Amigorena S, Raposo G, Clayton A (2006). Isolation and characterization of exosomes from cell culture supernatants and biological fluids. Curr Protoc Cell Biol.

[25] Zhou W, Fong MY, Min Y, Somlo G, Liu L, Palomares MR, Yu Y, Chow A, O'Connor ST, Chin AR (2014). Cancer-secreted miR-105 destroys vascular endothelial barriers to promote metastasis. Cancer Cell.

[26] Alvarez-Erviti L, Seow Y, Yin H, Betts C, Lakhal S, Wood MJ (2011). Delivery of siRNA to the mouse brain by systemic injection of targeted exosomes. Nat Biotechnol.

[27] Tian Y, Li S, Song J, Ji T, Zhu M, Anderson GJ, Wei J, Nie G (2014). A doxorubicin delivery platform using engineered natural membrane vesicle exosomes for targeted tumor therapy. Biomaterials.

[28] Wu WJ, Zhang Y, Zeng ZL, Li XB, Hu KS, Luo HY, Yang J, Huang P, Xu RH (2013). beta-phenylethyl isothiocyanate reverses platinum resistance by a GSH-dependent mechanism in cancer cells with epithelial-mesenchymal transition phenotype. Biochem Pharmacol.

[29] Fang T, Lv H, Lv G, Li T, Wang C, Han Q, Yu L, Su B, Guo L, Huang S (2018). Tumor-derived exosomal miR-1247-3p induces cancer-associated fibroblast activation to foster lung metastasis of liver cancer. Nat Commun.

[30] Yang MH, Hsu DS, Wang HW, Wang HJ, Lan HY, Yang WH, Huang CH, Kao SY, Tzeng CH, Tai SK (2010). Bmi1 is essential in Twist1-induced epithelial-mesenchymal transition. Nat Cell Biol.

[31] Wilson PM, Danenberg PV, Johnston PG, Lenz HJ, Ladner RD (2014). Standing the test of time: targeting thymidylate biosynthesis in cancer therapy. Nat Rev Clin Oncol.

[32] DeGorter MK, Xia CQ, Yang JJ, Kim RB (2012). Drug transporters in drug efficacy and toxicity. Annu Rev Pharmacol Toxicol.

[33] Ciafre SA, Galardi S, Mangiola A, Ferracin M, Liu CG, Sabatino G, Negrini M, Maira G, Croce CM, Farace MG (2005). Extensive modulation of a set of microRNAs in primary glioblastoma. Biochem Biophys Res Commun.

[34] Santos MC, Tegge AN, Correa BR, Mahesula S, Kohnke LQ, Qiao M, Ferreira MA, Kokovay E, Penalva LO (2016). miR-124, −128, and −137 orchestrate neural differentiation by acting on overlapping gene sets containing a highly connected transcription factor network. Stem Cells.

[35] Koh H, Park H, Chandimali N, Huynh DL, Zhang JJ, Ghosh M, Gera M, Kim N, Bak Y, Yoon DY (2017). MicroRNA-128 suppresses paclitaxel-resistant lung cancer by inhibiting MUC1-C and BMI-1 in cancer stem cells. Oncotarget.

[36] Kreso A, van Galen P, Pedley NM, Lima-Fernandes E, Frelin C, Davis T, Cao L, Baiazitov R, Du W, Sydorenko N (2014). Self-renewal as a therapeutic target in human colorectal cancer. Nat Med.

[37] Zhang X, Yang X, Zhang Y, Liu X, Zheng G, Yang Y, Wang L, Du L, Wang C (2015). Direct serum assay for cell-free bmi-1 mRNA and its potential diagnostic and prognostic value for colorectal cancer. Clin Cancer Res.

[38] Nies AT, Magdy T, Schwab M, Zanger UM (2015). Role of ABC transporters in fluoropyrimidine-based chemotherapy response. Adv Cancer Res.

[39] Oguri T, Isobe T, Suzuki T, Nishio K, Fujiwara Y, Katoh O, Yamakido M (2000). Increased expression of the MRP5 gene is associated with exposure to platinum drugs in lung cancer. Int J Cancer.

[40] Krutzfeldt J, Rajewsky N, Braich R, Rajeev KG, Tuschl T, Manoharan M, Stoffel M (2005). Silencing of microRNAs in vivo with ‘antagomirs’. Nature.

[41] Srinivasan S, Selvan ST, Archunan G, Gulyas B, Padmanabhan P (2013). MicroRNAs -the next generation therapeutic targets in human diseases. Theranostics.

[42] Li Y, Zheng Q, Bao C, Li S, Guo W, Zhao J, Chen D, Gu J, He X, Huang S (2015). Circular RNA is enriched and stable in exosomes: a promising biomarker for cancer diagnosis. Cell Res.

[43] Zhang Y, Liu D, Chen X, Li J, Li L, Bian Z, Sun F, Lu J, Yin Y, Cai X (2010). Secreted monocytic miR-150 enhances targeted endothelial cell migration. Mol Cell.

[44] van der Meel R, Fens MH, Vader P, van Solinge WW, Eniola-Adefeso O, Schiffelers RM (2014). Extracellular vesicles as drug delivery systems: lessons from the liposome field. J Control Release.

[45] Vader P, Mol EA, Pasterkamp G, Schiffelers RM (2016). Extracellular vesicles for drug delivery. Adv Drug Deliv Rev.

[46] Johnsen KB, Gudbergsson JM, Skov MN, Pilgaard L, Moos T, Duroux M (1846). A comprehensive overview of exosomes as drug delivery vehicles - endogenous nanocarriers for targeted cancer therapy. Biochim Biophys Acta.

[47] Brown EJ, Frazier WA (2001). Integrin-associated protein (CD47) and its ligands. Trends Cell Biol.

[48] Jaiswal S, Jamieson CH, Pang WW, Park CY, Chao MP, Majeti R, Traver D, van Rooijen N, Weissman IL (2009). CD47 is upregulated on circulating hematopoietic stem cells and leukemia cells to avoid phagocytosis. Cell.

[49] Kamerkar S, LeBleu VS, Sugimoto H, Yang S, Ruivo CF, Melo SA, Lee JJ, Kalluri R (2017). Exosomes facilitate therapeutic targeting of oncogenic KRAS in pancreatic cancer. Nature.

[50] Simoes S, Filipe A, Faneca H, Mano M, Penacho N, Duzgunes N, de Lima MP (2005). Cationic liposomes for gene delivery. Expert Opin Drug Deliv.

[51] Ursula A, Jana J, Katarina B, Petra P, Martin P, Pavel P, Ondrej T, Juraj K, Martina Z, Vanda R, Cestmir A. Prodrug suicide gene therapy for cancer targeted intracellular by mesenchymal stem cell exosomes. Int J Cancer. 2018. 10.1002/ijc.31792.10.1002/ijc.3179230098225

[52] Zhang X, Yuan X, Shi H, Wu L, Qian H, Xu W (2015). Exosomes in cancer: small particle, big player. J Hematol Oncol.

[53] O'Loughlin AJ, Woffindale CA, Wood MJ (2012). Exosomes and the emerging field of exosome-based gene therapy. Curr Gene Ther.

[54] Meyerhardt JA, Mayer RJ (2005). Systemic therapy for colorectal cancer. N Engl J Med.

